# Curative Effect Observation of Applying Silver-Zinc Bacteriostatic Cream to Patients with Second-Degree Burn under Targeted Nursing Intervention and Its Effect on Wound Healing Rate

**DOI:** 10.1155/2021/7591959

**Published:** 2021-12-08

**Authors:** Bingqing Li, Kun Xu, Xin Liu

**Affiliations:** Department of Burn and Plastic Surgery, Qingdao Municipal Hospital, Qingdao 266011, China

## Abstract

Second-degree burn is the most common type of burn wound in the clinics, which presents a deeper wound, skin blisters, white or red bottom, and thick and clear fluid inside, is sensitive to tenderness, and turns white by compression [1, 2]. The aim of this study is to explore the efficacy of applying silver-zinc bacteriostatic cream to patients with second-degree burn under targeted nursing intervention and its effect on wound healing rate. A total of 110 patients with second-degree burn treated in our hospital from January 2019 to June 2021 were selected as the research object for the retrospective study. Between the experimental group and the control group, no statistical differences in patients' general information were observed (*P* > 0.05); 1 week, 2 weeks, and 3 weeks after treatment, the visual analogue scale (VAS) pain scores of the experimental group were significantly lower (*P* < 0.05); and the total incidence rate of adverse reactions was remarkably lower in the experimental group (*P* < 0.05). On the basis of targeted nursing intervention, applying silver-zinc bacteriostatic cream obtains an obviously better clinical efficacy than silver sulfadiazine ointment in treating second-degree burn and works better in promoting wound healing, relieving pain sensation, and reducing adverse reactions.

## 1. Introduction

Second-degree burn is the most common type of burn wound in the clinics, which presents a deeper wound, skin blisters, white or red bottom, and thick and clear fluid inside, is sensitive to tenderness, and turns white by compression [1, 2]. The depth of burn can be divided into superficial second-degree burn and deep second-degree burn. In case of second-degree burn, the patients' dermis will be compromised, with necrotic tissue and exudate on the wound at the same time, the damaged skin loses the barrier against bacterial invasion, so the bacteria are prone to colonize the wound to initiate infection, followed by the coagulation and necrosis of parabiosis tissue on the surface, delay wound healing, and aggravation of scar hyperplasia after healing, and in severe cases, there will even have irreversible consequences [3–6]. In view of the severity and specificity of burn patients and to guarantee the therapeutic effect, the targeted nursing intervention centered on both nursing and treatment was implemented in our hospital to comprehensively promote the nursing quality for burn patients and obtain high nursing satisfaction. From the perspective of wound therapy, silver sulfadiazine is a classical choice for the treatment of burn wounds, but its poor stability, susceptibility to deterioration when exposed to light or heat, and chemical irritation and inert effects on the wound surface make it limited in clinical applications. With the continuous development of the pharmaceutical industry nowadays, many scholars have gradually recognized the value of silver agents in the treatment of burns. However, recent research at home and abroad on the efficacy of silver-zinc cream in the treatment of burns is still in the active exploration stage, with few related reports. Therefore, the comprehensive treatment program of applying silver-zinc bacteriostatic cream under the targeted nursing intervention for patients with the second-degree burn was implemented in our hospital without delaying the patients' condition, which obtained a better clinical efficacy and is summarized and reported as follows.

## 2. Materials and Methods

### 2.1. Patients Screening and Grouping

A total of 110 patients with second-degree burn treated in our hospital from January 2019 to June 2021 were selected as the research object for the retrospective study. The targeted nursing intervention was conducted to all patients, and according to the treatment methods, the patients were divided into the control group (silver sulfadiazine ointment treatment, *n* = 55) and the experimental group (silver-zinc bacteriostatic cream treatment, *n* = 55). The study was approved by the hospital ethics committee.

### 2.2. Inclusion Criteria

The inclusion criteria for patients were as follows. The clinical diagnosis criteria for second-degree burn were met [7]. The patients were 18–45 years old. The patients visited the hospital for the first time and did not conduct any treatments to the wound before admission. The patients' information were complete. The patients and their family members agreed to join the study and signed the informed consent.

### 2.3. Exclusion Criteria for Patients

The exclusion criteria for patients were as follows. Presence of other severe organic diseases, malignant tumors, or coagulation disorders. Long-term malnutrition. Allergy to or development of severe adverse reactions from silver-zinc bacteriostatic cream. Presence of immunological diseases, hematological diseases, or acute metabolic disorder. Allergy to silver, zinc, and sulfa drugs. Pregnant or lactating patients.

### 2.4. Methods

The steps of targeted nursing intervention were as follows. (1) After admission, the patients' wounds were cleaned immediately, i.e., first flushing the wound with normal saline, then repeatedly cleaning it with diluted hydrogen peroxide aqueous solution three times, wiping the wound, and disinfecting with povidone-iodine solution for 3 min, and treatments such as fluid infusion and analgesia were performed [8–10]. (2) The targeted mental intervention was performed, including communicating with patients or their family members in a timely manner to understand the differences in the mental state of patients, asking for information about patients' family data, etiological factors of burn, and social support to find out the reason for poor mental state of patients, and providing targeted psychological guidance to obtain the emotional support from the patients' family members and promote the patients' confidence in treatment and compliance. (3) The targeted environmental nursing was implemented. Patients with wound pain might have symptoms such as insomnia, so the nursing personnel should optimize the ward environment as much as possible according to the patients' condition, including adjusting the humidity, temperature, and light, paying attention to the ward hygiene and ensuring a quiet ward to reduce the irritation from poor environment. In addition, the nursing personnel could play proper light music in the ward according to the patients' preferences or provide newspapers, audio books, and other materials to distract their attention [11–14]. (4) The targeted health education was implemented. With the difference between individuals, patients differed in their degree of awareness of the disease, so the nursing personnel should carry out targeted education on patients according to their age and educational degree, informed the patients about the daily precautions, possible complications, and prevent and control measures in detail based on their specific condition, and ensured that the education contents were clear and the education approach was appropriate. (5) The targeted complications nursing was implemented. Special attention was paid to the nursing of patients' mouth cavity, respiratory tract, gastrointestinal tract, and urinary system, the preventive measures for infection were carried out, and the patients' autoimmunity was improved by reasonable diet to avoid complications as much as possible [11, 15, 16].

For patients in the control group, the wound was applied with the proper amount of silver sulfadiazine ointment (specification: 500 g/tube; manufactured: Zhejiang Hacon Pharmaceutical Co., Ltd.; NMPA approval no. H33020325) for 1.5 mm thick and then covered and fixed with sterile gauze, and the fresh dressing was changed once in one or two days. For patients in the experimental group, the wound was applied with silver-zinc bacteriostatic cream prepared by our hospital (5% of sulfadiazine zinc and 1% of sulfadiazine silver) for 1.5 mm thick and then covered and fixed with sterile gauze, and the fresh dressing was changed once in one or two days. The time of medication was decided according to the patients' condition.

### 2.5. Observation Indexes

The general information mainly included the patients' age, gender, etiological factors of burn, depth of burn, and burn position. The observation indexes for basic clinical situation mainly included the time of antibiotic treatment, hospitalization time, and wound healing time (i.e., the time of complete epithelization of wound).

Wound healing rate = (initial wound area – wound area after treatment)/initial wound area × 100%. To calculate the area, the wound was fully covered with sterile plastic film to get the contour and then scan to the computer.

The proper amount of secretions on the patients' wounds was taken by sterile throat swab and sent to the laboratory department of our hospital for bacterial culture, and the positive cases were counted. The pain intensity of wound was evaluated by the visual analogue scale (VAS) on a scale of 0–10, with 0 points indicating no pain and 10 points indicating unbearable severe pain. According to the examination results of indicators such as routine blood tests and hepatic and kidney function and combined with the clinical manifestation, the incidence of adverse reactions in patients was evaluated.

### 2.6. Statistical Processing

In this study, the between-group differences in data were processed by SPSS 22.0, the picture drawing software was GraphPad Prism 7 (GraphPad Software, San Diego, USA), items included were enumeration data and measurement data, which were expressed by (*n*(%)) and ($\bar{x}$ ± s) and examined by the *X*^2^ test and *t*-test, respectively, and differences were considered statistically significant at *P* < 0.05.

## 3. Results

### 3.1. General Information

No statistical differences in patients' general information were observed (*P* > 0.05), which met the criteria for the controlled study (Table 1).

### 3.2. Basic Clinical Performance

The time of antibiotic treatment, hospitalization time, and wound healing time of patients were significantly shorter in the experimental group than in the control group (*P* < 0.05) (Figure 1).

### 3.3. Wound Healing Rate

From day 3 to day 21 of treatment, the wound healing rates of superficial and deep second-degree burn patients were significantly higher in the experimental group than in the control group (*P* < 0.05) (Table 2).

### 3.4. Results of Wound Bacterial Culture

One week and two weeks after treatment, the positive rates of bacterial culture were significantly lower in the experimental group than in the control group (*P* < 0.05), and at the 3^rd^ week, the positive rate of the experimental group was 0, which was lower than the control group, but with no significant between-group difference (*P* > 0.05) (Figure 2).

### 3.5. VAS Pain Scores

One week, two weeks, and three weeks after treatment, the VAS pain scores of patients were significantly lower in the experimental group than in the control group (*P* < 0.05) (Table 3).

### 3.6. Adverse Reactions

The total incidence rate of adverse reactions was significantly lower in the experimental group than in the control group (*P* < 0.05) (Figure 3).

## 4. Discussion

Silver sulfadiazine has been a classic topical drug used in the clinics to treat burn wounds. It mainly contains sulfadiazine and silver ion, so it has the antibacterial action of sulfadiazine and the astringency of silver salt and a powerful inhibitory effect on both Gram-positive coccus and Gram-negative bacillus [17–20]. But long-term clinical application exposes many disadvantages of silver sulfadiazine. First, long-term use greatly increases the drug resistance of bacteria, which is directly manifested by reduced bactericidal ability; second, the drug has a high content of silver ion, which will bind to RNA of epithelial cells and is not conducive to epithelial cell regeneration; as a whole, the drug can irritate the wounds and is unfavorable to wound repair; finally, it not only has poor stability but also easily leads to many adverse reactions and complications such as granulocytopenia and thrombocytopenia, aplastic anemia, and liver dysfunction. Second-degree burn has been the focus of clinical treatment, especially the deep second-degree burn. Patients who suffer from deep second-degree burn have obvious tissue necrosis on the wound and wound exudation and are susceptible to infection [21–23]. The main reason affecting the wound healing of the second-degree burn is that the early vascular stasis band turns into a coagulation necrosis band under the impact of bacterial infection, which subsequently leads to the necrosis of the parabiosis tissue, resulting in delayed wound healing and aggravated scar hyperplasia. On the other hand, wound environmental care during the treatment process is also an important aspect that affects the outcome of patients. Therefore, from the viewpoint of comprehensive treatment, the targeted nursing intervention was conducted for patients with second-degree burn treated in our hospital to guarantee clinical efficacy. However, how to improve the rate of wound epithelialization and inhibit bacterial growth and reproduction is still the key to the treatment of second-degree burn.

By summarizing and analyzing the previous research experience, the advantages and disadvantages of the existing silver preparations for the treatment of burn wounds have been clarified, so the silver-zinc bacteriostatic cream made by our hospital was used for treating patients with second-degree burn, which obtained a better efficacy, with the results concluded as follows. The time of antibiotic treatment, hospitalization time, and wound healing time of patients were significantly shorter in the experimental group than in the control group (*P* < 0.05), and from day 3 to day 21 of treatment, the wound healing rates of superficial and deep second-degree burn patients were significantly higher in the experimental group than in the control group (*P* < 0.05). Compared with the study conducted by Quang Hieu Tran et al. [24], the wound healing time obtained by the control group of this study was obviously shortened, indicating that the targeted nursing intervention might promote wound healing, and the observation indicators of the experimental group were improved remarkably, proving that in terms of promoting wound healing and reducing the use of antibiotics, silver-zinc bacteriostatic cream worked better than silver sulfadiazine ointment because the silver ion and zinc ion in the silver-zinc bacteriostatic cream could effectively reduce wound exudation, promote wound drying and astringency, and prevent body fluid loss. In addition, after 1 week and 2 weeks of treatment, the positive rates of bacterial culture were significantly lower in the experimental group than in the control group (*P* < 0.05), and at the 3^rd^ week, the positive rate of the experimental group was 0, which was lower than the control group, but with no significant between-group difference (*P* > 0.05), demonstrating that both silver sulfadiazine and silver-zinc bacteriostatic cream had the antibacterial effect, but the latter worked faster and reduced the irritation of silver sulfadiazine on wounds. Compared with the control group, the VAS pain scores of patients after 1 week, 2 weeks, and 3 weeks of treatment of the experimental group were significantly lower (*P* < 0.05); and the total incidence rate of adverse reactions was significantly lower in the experimental group than in the control group (*P* < 0.05), proving that silver-zinc bacteriostatic cream could protect the burn wounds and prevent excessive evaporation of water, cell dehydration, and tissue fracture, thereby, reducing the pain sensation for patients. Although the adverse reaction rate of silver-zinc bacteriostatic cream is lower, attention should be paid to the prevention and treatment of adverse reactions such as wound deepening and high fever, which can be reduced by strengthening targeted nursing intervention for adverse reactions.

## 5. Conclusion

In conclusion, on the basis of targeted nursing intervention, applying silver-zinc bacteriostatic cream obtains an obviously better clinical efficacy than silver sulfadiazine ointment in treating second-degree burn and works better in promoting wound healing, relieving pain sensation, and reducing adverse reactions. But this study still has the following problems. It was a single center pharmaceutical study, and the sample size was small because of the limited cost of analysis. The long-term follow-up mechanism was not established for the patients, and thus, long-term efficacy analysis of topical medication was lacking.

## Figures and Tables

**Figure 1:** Analysis of patients' basic clinical performance. The horizontal axis indicates the evaluation indicators, and the vertical axis indicates the number of days (d). The time of antibiotic treatment, hospitalization time, and wound healing time of the control group were (6.35 ± 1.47), (16.63 ± 2.52), and (18.47 ± 2.51), respectively. The time of antibiotic treatment, hospitalization time, and wound healing time of the experimental group were (11.94 ± 3.42), (22.83 ± 2.14), and (26.88 ± 6.74), respectively. ^*∗*^Difference in time of antibiotic treatment between the two groups was significant (*t* = 11.137, *P* < 0.001). ^*∗∗*^Difference in hospitalization time between the two groups was significant (*t* = 13.908, *P* < 0.001). ^*∗∗∗*^Difference in wound healing time between the two groups was significant (*t* = 8.672, *P* < 0.001).

**Figure 2:** Positive rate of wound bacterial culture (*n* = 55, %). The horizontal axis indicates the time points of bacterial culture, and the vertical axis indicates the positive rate (%). Before treatment and 1 week, 2 weeks, and 3 weeks after treatment, the numbers of positive cases in the control group were 28, 19, 12, and 2, respectively. Before treatment and 1 week, 2 weeks, and 3 weeks after treatment, the numbers of positive cases in the experimental group were 27, 9, 4, and 0, respectively. ^*∗*^1 week after treatment, the difference in positive rate between the two groups was significant (*X*^2^ = 4.791, *P*=0.029). ^*∗∗*^2 weeks after treatment, the difference in positive rate between the two groups was significant (*X*^2^ = 4.681, *P*=0.031).

**Figure 3:** Adverse reactions (*n* = 55, %). The horizontal axis indicates the adverse reactions, and the vertical axis indicates the incidence rate (%). A total of 10 patients in the control group had adverse reactions, including 3 cases with wound deepening, 4 cases with wound odor, and 3 cases with high fever. A total of 3 patients in the experimental group had adverse reactions, including 1 case with wound deepening and 2 cases with high fever. ^*∗*^Difference in the total incidence rate of adverse reactions between the two groups was significant (*X*^2^ = 4.274, *P*=0.039).

**Table 1:** Patients' general information (*n* = 55).

Observation indicator	Control group	Experimental group	*X* ^2^/*t*	*P*
Age (years)	36.37 ± 6.15	37.25 ± 5.76	0.708	0.481
Gender			0.202	0.654
Male	41 (74.55)	43 (78.18)		
Female	14 (25.45)	12 (21.82)		
Etiological factor of burn				
Fire	34 (61.82)	32 (58.18)	0.152	0.697
Boiling liquid	11 (20)	13 (23.64)	0.213	0.644
Chemical	6 (10.91)	7 (12.73)	0.087	0.768
Others	4 (7.27)	3 (5.45)	0.153	0.696
Burn degree			0.161	0.688
Superficial second-degree burn	35 (63.64)	37 (67.27)		
Deep second-degree burn	20 (36.36)	18 (32.73)		
Proportion of burn (%)	11.84 ± 4.07	12.25 ± 4.41	0.507	0.613
BMI (kg/m^2^)	23.84 ± 3.26	23.77 ± 3.37	0.111	0.912
Burn position				
Face	26 (47.27)	28 (50.91)	0.146	0.703
Chest	21 (38.18)	19 (34.55)	0.157	0.692
Upper limb	33 (60)	36 (65.45)	0.350	0.554
Lower limb	22 (40)	25 (45.45)	0.334	0.563

**Table 2:** Patients' wound healing rate (%).

Time	Control group (*n* = 55)		Experimental group (*n* = 55)	
	Superficial second-degree	Deep second-degree	Superficial second-degree	Deep second-degree
Day 3	37.84 ± 5.22^*∗*^	33.64 ± 5.51^*∗*^	49.07 ± 3.82	43.97 ± 5.46
Day 7	64.15 ± 7.32^*∗*^	57.74 ± 7.35^*∗*^	79.01 ± 7.93	72.25 ± 6.90
Day 14	74.91 ± 8.07^*∗*^	69.98 ± 7.78^*∗*^	86.13 ± 8.81	84.23 ± 8.82
Day 21	83.52 ± 8.11^*∗*^	80.64 ± 8.20^*∗*^	90.84 ± 9.08	88.85 ± 9.12

^*∗*^ *P* < 0.05 vs. the experimental group at the same time period.

**Table 3:** Analysis of patients' VAS pain scores.

Group	Before treatment	1 week after treatment	2 weeks after treatment	3 weeks after treatment
Control	9.15 ± 1.50	7.25 ± 1.53	5.94 ± 1.91	3.12 ± 1.21
Experimental	9.47 ± 1.46	6.07 ± 1.32	4.05 ± 1.35	2.03 ± 1.07
*t*		4.331	5.993	5.005
*P*		<0.001	<0.001	<0.001

## Data Availability

The datasets used and/or analyzed during the current study are available from the corresponding author upon request.
